# Characterizing the immune response of chickens to *Campylobacter jejuni* (Strain A74C)

**DOI:** 10.1371/journal.pone.0247080

**Published:** 2021-03-15

**Authors:** Mohamad Mortada, Douglas E. Cosby, Gabriel Akerele, Nour Ramadan, Jarred Oxford, Revathi Shanmugasundaram, Theros T. Ng, Ramesh K. Selvaraj

**Affiliations:** 1 Department of Poultry Sciences, The University of Georgia, Athens, Georgia, United States of America; 2 USDA-ARS, Poultry Microbiological Safety and Processing Research Unit, Athens, Georgia, United States of America; 3 USDA-ARS, Toxicology and Mycotoxin Unit, Athens, Georgia, United States of America; USDA-Agricultural Research Service, UNITED STATES

## Abstract

*Campylobacter* is one of the major foodborne pathogens causing bacterial gastroenteritis worldwide. The immune response of broiler chickens to *C*. *jejuni* is under-researched. This study aimed to characterize the immune response of chickens to *Campylobacter jejuni* colonization. Birds were challenged orally with 0.5 mL of 2.4 x 10^8^ CFU/mL of *Campylobacter jejuni* or with 0.5 mL of 0.85% saline. *Campylobacter jejuni* persisted in the ceca of challenged birds with cecal colonization reaching 4.9 log10 CFU/g on 21 dpi. *Campylobacter* was disseminated to the spleen and liver on 7 dpi and was cleared on 21 dpi from both internal organs. Challenged birds had a significant increase in anti-*Campylobacter* serum IgY (14&21 dpi) and bile IgA (14 dpi). At 3 dpi, there was a significant suppression in T-lymphocytes derived from the cecal tonsils of birds in the challenge treatment when compared to the control treatment after 72 h of *ex vivo* stimulation with Con A or *C*. *jejuni*. The T-cell suppression on 3 dpi was accompanied by a significant decrease in LITAF, K60, CLAU-2, IL-1β, iNOS, and IL-6 mRNA levels in the ceca and an increase in nitric oxide production from adherent splenocytes of challenged birds. In addition, on 3 dpi, there was a significant increase in CD4+ and CD8+ T lymphocytes in the challenge treatment. On 14 dpi, both pro and anti-inflammatory cytokines were upregulated in the spleen, and a significant increase in CD8+ T lymphocytes in *Campylobacter*-challenged birds’ ceca was observed. The persistence of *C*. *jejuni* in the ceca of challenged birds on 21 dpi was accompanied by an increase in IL-10 and LITAF mRNA levels, an increase in MNC proliferation when stimulated *ex-vivo* with the diluted *C*. *jejuni*, an increase in serum specific IgY antibodies, an increase in both CD4+ and CD8+ cells, and a decrease in CD4+:CD8+ cell ratio. The balanced Th1 and Th2 immune responses against *C*. *jejuni* might explain the ceca’s bacterial colonization and the absence of pathology in *Campylobacter*-challenged birds. Future studies on T lymphocyte subpopulations should elucidate a pivotal role in the persistence of *Campylobacter* in the ceca.

## Introduction

*Campylobacter* is one of the major foodborne pathogens that cause bacterial gastroenteritis worldwide [1]. The economic burden of campylobacteriosis, that includes direct and indirect costs, is estimated to be around $2 billion [2]. Most campylobacteriosis cases are caused mainly by *C*. *jejuni*, and are attributed to handling and consumption of raw or undercooked poultry meat [3, 4]. *Campylobacter jejuni* is considered to be one of the commensal microorganisms in the avian gut recovered from a wide range of domestic poultry [5]. However, many researchers are presenting evidence that *Campylobacter* is not merely a commensal and but is capable of inducing a pro-inflammatory response and affect broilers’ performance parameters [6, 7].

*Campylobacter* colonization is highly prevalent in commercial broiler flocks. A study showed that 95% of birds could be rapidly colonized with *Campylobacter*, once exposed to a single infected seeder bird, and remain colonized until market age [8]. Most commercial broiler flocks remain *Campylobacter*-negative until 2-wk of age. This early protection has been attributed to maternally-derived antibodies [9]. *Campylobacter* colonizes the ceca primarily where the bacterial load can reach up to 10^9^ CFU/g [9]. Even though *Campylobacter* is considered as commensal, researchers have shown that *Campylobacter jejuni* can disseminate to internal organs, namely the spleen, liver/gallbladder, thymus, and bursa of Fabricius as early as 1 h, 1 day, and 1 wk post-infection [10].

The immune response of broilers to *Campylobacter* colonization and the factors responsible for *Campylobacter* persistence in the chicken gut are not well characterized [1]. Many researchers suggest that *Campylobacter* could induce a pro-inflammatory response such as the upregulation of IL-1β, and could affect body weight gain by reducing nutrient absorption and competing for amino acids in the gut [7, 11]. However, other researchers showed an upregulation in IL-10 regulatory cytokine seen as a breed-dependent response in colonization when comparing fast versus slow-growing breeds [6].

Recently, the American Association for Avian Pathologists has listed the reduction of *Campylobacter* in poultry as one of the top research priorities for 2019. In addition, one of the main challenges facing poultry processors in the US is compliance with the new *Campylobacter* standards set by USDA-FSIS [12]. We believe that understanding the immune response of broilers to *Campylobacter* colonization is a prerequisite for evaluating or developing any successful intervention [1]. Therefore, this study aimed to characterize the immune response of broilers to *Campylobacter jejuni* (Strain A74C) [13–15] and help elucidate the immune responses that are responsible for the highly colonizing nature of *Campylobacter jejuni*. To our knowledge this is the first study that evaluates the effect of *C*. *jejuni* on the proliferation of T lymphocytes and their CD4+ and CD8+ populations.

## Materials and methods

### Ethics statement

All animal protocols were approved by the Institutional Animal Care and Use Committee at the University of Georgia (AUP: A2018 04-010-Y2-A2). Researchers involved in the *in vivo* trial were trained by the University of Georgia on animal care and handling (UGA IACUC 101 course). Birds were monitored at least once a day for lethargy, loss of body weight, ruffled feathers, diarrhea, and dehydration during the *in vivo* experiment. Birds that could not move or refused to eat were immediately humanely euthanized by cervical dislocation. None of the birds were found dead during this trial and two birds reached the humane endpoint and were immediately humanely euthanized. Birds were euthanized during sampling timepoints and the last day of the study (day 35).

### Birds and *Campylobacter jejuni* challenge

A total of 240 day-old broiler chicks was co-mingled and raised until d14. On d14, broilers were randomly assigned to two treatments, control, and challenge, with 20 birds per cage and six cages per treatment (n = 6). Birds in the two treatments were weight-matched, and cage weights were normalized to a mean body weight of 409g/bird/cage (LL:329*g* and UL: 489*g*). After weigh-matching, birds from the two treatments were placed in two identical BSL-2 rooms at the Poultry Research Center at The University of Georgia. Birds were orally challenged with 0.5 mL of 2.4 x 10^8^ CFU/mL of *Campylobacter jejuni* or with 0.5 mL of 0.85% saline. All birds were fed a corn and soybean meal diet during co-mingling (d0-d14) and throughout the trial period d14—d35 (Table 1). Three birds per cage were euthanized by cervical dislocation and ceca, cecal tonsil, spleen, liver, blood, and bile were collected on the day of challenge (0 dpi), 1, 3, 7, 14, and 21 dpi for microbiological and immunological parameters. Body weight and feed consumption were recorded weekly, and body weight gain and feed conversion ratio were analyzed. The FCR was corrected for bird removals and mortality.

**Table 1:** Basal diet ingredients and calculated nutrient composition.

	Starter (0 –d 35)
Ingredients	%
Corn	58.47
Soybean Meal, 48% CP	35.15
Soybean Oil	2.27
Monocalcium phosphorus, 21%	1.38
Limestone	1.59
DL-Methionine	0.21
L-Lysine-HCL, 78%	0.14
Salt (NaCl)	0.35
Vitamin premix^1^	0.08
Mineral premix^2^	0.35
Total:	100.0
Calculated Nutrient Composition	
ME, kcal/kg	3,050
Crude Protein, %	21.44
Crude Fat, %	4.55
Crude Fiber, %	2.17
Calcium, %	0.95
Total Phosphorus, %	0.71
Avail. Phosphorus< %	0.45
Sodium, %	0.16
Potassium, %	0.92
Chloride, %	0.27
Lysine, %	1.31
Methionine, %	0.56
TSAA, %	0.91
Threonine, %	0.87
Tryptophan, %	0.29
Arginine, %	1.50

^1^ Vitamin mix provided the following (per kilogram of diet): thiamin-mononitrate, 2.4 mg; nicotinic acid, 44 mg; riboflavin, 4.4 mg; D-Ca pantothenate, 12 mg; vitamin B12 (cobalamin), 12.0g; pyridoxine-HCl, 2.7 mg; D-biotin, 0.11 mg; folic acid, 0.55 mg; menadione sodium bisulfate complex, 3.34 mg; choline chloride, 220 mg; cholecalciferol, 1,100 IU; trans-reinyl acetate, 2,500 IU; all-rac-tocopherol acetate, 11 IU; ethoxyquin, 150 mg.

^2^ Trace mineral mix provides the following (per kilogram of diet): manganese (MnSO4.H2O), 101 mg; iron (FeSO4.7H2O), 20 mg; zinc (Zn)), 80 mg; copper (CuSO4.5H2O), 3 mg; iodine (ethylene diamine dihydroiodide), 0.75 mg; magnesium (MgO), 20 mg; selenium (sodium selenite), 0.3 mg.

### *Campylobacter jejuni* challenge

*Campylobacter jejuni* (Strain A74C) previously studied by [13–15] was propagated on Campy-CEFEX agar and incubated for 48 h in a microaerobic atmosphere (85% N_2_, 10% CO_2_, and 5% O_2_) at 42°C. After incubation, bacterial cells were harvested using sterile cotton swabs and resuspended in 0.85% saline (NaCl, Sigma Chemical Co., St. Louis, MO) to create a suspension with an optical density of 0.20 at 540nm with a Spec-20 (Milton-Roy Spectrophotometer, Thermo Spectronics, Madison, WI). This optical density value is equivalent to 2 x 10^8^ CFU/mL of *Campylobacter* [16]. The challenge stock, 2.4 x 10^8^ CFU/mL of *C*. *jejuni* A74C, was confirmed by serial dilutions and direct plating on Campy-CEFEX.

### Effect of *Campylobacter jejuni* challenge on *Campylobacter* load in the ceca, spleen, and liver

On 7, 14, and 21 dpi, ceca, spleen, and liver were dissected, and a total of 108 samples (3 birds/cage x 6 cages/treatment x 2 treatments x 3 organs) were aseptically collected into stomacher bags, placed on ice, and transported to the laboratory. Samples were macerated with a rubber mallet, and 3X (wt/vol) 1X Bolton’s broth supplemented with Bolton selective supplements (HiMedia Laboratories, West Chester, PA) were added, and bags were stomached for 60 s. A volume of 10 μl of homogenates was directly plated or serially diluted in 7 tubes having 90ul of 0.85% saline resulting in 10^−1^ to 10^−8^ dilutions using the microdilutions method as described by [12]. From every dilution, a volume of 10μl was spotted in triplicate on campy-CEFEX agar. Plates were then incubated for 48 h in a microaerobic atmosphere at 42°C. After incubation, colonies were counted and confirmed by microscopic observation for characteristic cork-screw morphology and motility on wet mount preparations. Colonies were further confirmed using SyBr green qPCR and primers targeting *C*. *jejuni mapA* gene (Table 2). Enumeration data were recorded as CFU/g and then transformed to log10 CFU/g for statistical analysis.

**Table 2:** Primers and PCR conditions for RTqPCR.

Target Gene	Sequence (5’-3’)	Annealing Temperature	Reference
IL-10-F	CATGCTGCTGGGCCTGAA	58.0°C	[22]
IL-10-R	CGTCTCCTTGATCTGCTTGATG		
TGF-β4 –F	CATACTCCTGGGTCTGGTTGGT	58.0°C	[23]
TGF-β4 –R	GACAGCCATCCGCATCTTCT		
TLR-4-F	ACCTACCCATCGGACACTTG	60.0°C	[24]
TLR-4-R	TGCCTGAGAGGTCAGGTT		
IL-1β-F	GCATCAAGGGCTACAAGCTC	58.0°C	[25]
IL-1β-R	CAGGCGGTAGAAGATGAAGC		
LITAF-F	ATCCTCACCCCTACCCTGTC	58.0°C	[26]
LITAF-R	GGCGGTCATAGAACAGCACT		
iNOS-F	AGTGGTATGCTCTGCCTGCT	60.0°C	[27]
iNOS-R	CCAGTCCCATTCTTCTTCC		
K60-F	ATTTCCTCCTGCCTCCTACA	55.0°C	[28]
K60-R	GTGACTGGCAAAAATGACTCC		
IL-6-F	CAAGGTGACGGAGGAGGAC	57.5°C	[29]
IL-6-R	TGGCGAGGAGGGATTTCT		
IL-4-F	AACATGCGTCAGCTCCTGAAT	57.5°C	[30]
IL-4-R	TCTGCTAGGAACTTCTCCATTGAA		
CLAU-2-F	CCTGCTCACCCTCATTGGAG	55.0°C	[31]
CLAU-2 R	GCTGAACTCACTCTTGGGCT		
ZO-1-F	TGTAGCCACAGCAAGAGGTG	55.0°C	[32]
ZO-1-R	CTGGAATGGCTCCTTGTGGT		
GAPDH -F	TCCTGTGACTTCAATGGTGA	55.0°C	[33]
GAPDH -R	CACAACACGGTTGCTGTATC		
*mapA*-F	CTGGTGGTTTTGAAGCAAAGATT	55.0°C	[34]
*mapA*-R	CAATACCAGTGTCTAAAGTGCGTTTAT		

### Effect of *Campylobacter jejuni* challenge on *Campylobacter jejuni mapA* gene in the ceca

On 0, 7, 14, and 21 dpi, ceca were dissected from three birds per cage and pooled aseptically into one stomacher bag/cage (n = 6), placed on ice, and transported to the laboratory. Ceca samples were macerated with a rubber mallet, and 3X (wt/vol) buffered peptone water was added. Samples were then stomached for 60 s, and ceca homogenates were stored at -80 °C. Bacterial DNA from the ceca was isolated, as described previously [17]. *Campylobacter jejuni* bacterial DNA in the ceca was quantified using SyBr green qPCR with primers targeting *C*. *jejuni mapA* gene (Table 2). Quantification data were reported as 40—Ct and then were statistically analyzed.

### Effect of *Campylobacter jejuni* challenge on serum IgY and bile IgA anti-*Campylobacter* antibodies

On 0d of age, blood was collected and pooled from 3 broiler chicks to measure the specific maternally derived serum anti-*Campylobacter* IgY antibodies. On 0, 7, 14, and 21 dpi, blood and bile were collected and pooled from 3 birds per cage. Specific serum IgY and bile IgA antibodies directed against *C*. *jejuni* (Strain A74C) whole-cell (WC) antigens were determined by enzyme-linked immunosorbent assay (ELISA) as described previously by [18] with modifications. Briefly, WC antigen was prepared by lysing 1X10^9^ CFU/ml of *C*. *jejuni* (Strain A74C) by seven cycles of bead-beating (TissueLyser LT, Qiagen, Germantown, MD) using acid-washed glass beads (Sigma-Aldrich, MO, USA) followed by freezing and thawing. ELISA plates (Nunc Maxisorp^™^, ThermoFisher Scientific, Waltham, MA) were coated with 2.5 μg/ml of WC diluted in coating buffer (carbonate/bicarbonate, pH 9.6). Serum was diluted 1:10 and bile was diluted 1:200 in PBS containing 2.5%, non-fat dry milk and 0.1% Tween 20 (VWR, Radnor, PA). The Horseradish peroxidase (HRP) conjugated polyclonal goat anti-chicken IgG (Bethyl, Montgomery, TX) and HRP-conjugated polyclonal goat anti-chicken IgA (SouthernBiotech, Birmingham, AL) were used at 1:10,000 as a secondary antibody. The absorbance was measured at 450 nm using Epoch microplate spectrophotometer (BioTek, VT, USA) and antibody levels were reported as OD 450 values.

### Effect of *Campylobacter jejuni* challenge on cecal tonsil CD4+ and CD8+ T lymphocytes, and CD4+:CD8+ cell ratio

On 0, 1, 3, 14, and 21 dpi, cecal tonsils from three birds per cage were aseptically pooled into a 5 mL tube having 3 mL of RPMI, placed on ice, and transported to the laboratory. Flow cytometry analysis for CD4+ and CD8+ cells was performed as described by [19]. Single-cell suspensions of the cecal tonsils (1 × 10^6^ cells) were incubated with PE-conjugated mouse anti-chicken CD4 and FITC-conjugated mouse anti-chicken CD8 (Southern Biotech, Birmingham, AL) at 1:200 dilution, and unlabeled mouse IgG at 1:500 dilution in a 96-well plate for 20 minutes. After incubation, cells were washed twice by centrifugation at 400 x g for 5 minutes using wash buffer (1× PBS, 2 mM EDTA, 1.5% FBS) to remove unbound primary antibodies. After washing, cells were analyzed using CytoSoft software (Guava Easycyte, Millipore, Billerica, MA). CD4+ and CD8+ cells were reported as the percentage of gated cells, and CD4+:CD8+ ratio was calculated.

### Effect of *Campylobacter jejuni* challenge on immune gene expression

On 0,1, 3, 7, 14, and 21 dpi cecal tonsil and spleen samples were dissected, and 3 organs per cage were pooled in 5 mL tubes filled with 3 ml of RNAlater (Qiagen, Germantown, MD). Samples were stored for seven days at 4°C until RNAlater permeated the tissue and stabilized the RNA. Excess RNAlater was removed from tubes, and samples were stored at -80°C until analyzed. Total RNA was extracted from cecal tonsils and reverse transcribed into cDNA [20]. The mRNA was analyzed for TGF-β4, IL-10, IL-1β, LITAF, TLR-4, iNOS, K60, IL-4, IL-6, CLAU-2, and ZO-1 genes by real-time PCR (CFX96 Touch Real Time System, BioRad) using SyBr green after normalizing for GAPDH mRNA (Table 2). The fold change from the reference was calculated using the 2^(Ct Sample—Housekeeping)^/2^(Ct Reference—Housekeeping)^ comparative Ct method, where Ct is the threshold cycle [21]. The Ct was determined by iQ5 software (Biorad) when the fluorescence rises exponentially 2-fold above the background.

### Effect of *Campylobacter jejuni* challenge on nitric oxide production from adherent splenocyte MNCs

On 1, 3, 7, 14, and 21 dpi, spleens were dissected from three birds per cage, and half-spleens were aseptically pooled into a 5 mL tube having 3 mL of RPMI, placed on ice, and transported to the laboratory. Spleens were strained using a 45μm cell strainer (Fisher scientific) to obtain a single-cell suspension. A volume of 3 mL of single-cell suspension was enriched for MNCs by density centrifugation over 3 mL of Histopaque (1.077 g/mL, Sigma-Aldrich, St. Louis, MO) for 10 min at 1,200 X g at 10°C without breaks as described by [35] with modifications. The splenocyte MNCs were washed and resuspended in 8 mL of complete RPMI-1640 medium (media supplemented with 4% FBS, 2% chicken serum, and 1% penicillin plus streptomycin) in T75 cell culture flasks and incubated in a 5% CO2 incubator at 42°C. After 24 h of incubation, non-adherent cells were washed with PBS, and adherent cells were removed by trypsinization (5 ml of 0.4% trypsin supplemented with 0.025% EDTA). Adherent cells were then washed in 20 mL of complete media and resuspended in 1 mL of complete RPMI for counting. Splenocyte MNCs were reseeded in triplicates in 96-well plates (100 μL/well of 5 x 10^5^ cells/mL). Cells were stimulated by adding a volume of 100 μL of complete RPMI media supplemented with 10 μg/mL of *Salmonella* Enteritidis LPS (Sigma Chemicals, MO, USA) or 20 μg/mL of lysed *C*. *jejuni* (Strain A74C). *Campylobacter jejuni* (Strain A74C) was lysed by seven cycles of bead-beating followed by freezing and thawing, as described above. The 96-well plates were then incubated for 48 h. After incubation, plates were centrifuged at 400 X g for 10 min, and the supernatant was removed. Nitrite levels in the supernatant were determined using the Griess method [36]. A volume of 100 μL of sulfanilamide/*N*-(1-Naphthyl) ethylenediamine dihydrochloride solution (#R2233500, Ricca Chemical Company, Arlington, TX) was added to 100 μl of the supernatant. After 5 min of incubation in the dark and at room temperature, absorbance was measured at 540 nm using Epoch microplate spectrophotometer (BioTek, VT, USA), and OD 540 values were recorded. The nitrite concentration in the samples was determined using the equation derived from the standard curve of serially diluted sodium nitrite Vs. OD 540 values.

### Effect of *Campylobacter jejuni* on the proliferation of cecal tonsil MNCs

On 1 and 3 dpi, cecal tonsils from three birds per cage were aseptically pooled into a 5 mL tube having 3 mL of RPMI, placed on ice, and transported to the laboratory. Cecal tonsil Mononuclear Cells (MNCs) were collected by straining the cecal tonsils for single-cell suspension using a 45μm cell strainer (Fisher scientific). The MNCs were then washed by centrifugation and resuspended in complete RPMI to a cell density of 5 x 10^5^ cells/mL. A volume of 100 μL of the cell suspension was added in triplicates to 96-well plates. Cecal tonsil mononuclear cells were then stimulated with complete RPMI media supplemented with Con A (15μg/mL) or 20 μg/mL of lysed *C*. *jejuni* (Strain A74C). The 96-well culture plates were then incubated for 72 h in a 5% CO2 incubator at 42°C. At 72 h of incubation, the proliferation of MNCs was measured using MTT tetrazolium 3-(4,5-dimethylthiazol-2-yl)-2,5-diphenyltetrazolium bromide) colorimetric assay as previously described [37], and obtained optical density values at 570nm (BioTek Epoch spectrophotometer; GEN5 3.03 software) were statistically analyzed.

### *Ex vivo* stimulation of cecal tonsil MNCs with lysed *C*. *jejuni* (Strain A74C) or *Salmonella* Enteritidis OMPs

To investigate the antigen-specific response of cecal tonsil mononuclear cells, on 7, 14, and 21 dpi, MNCs were seeded in 96-well plates in triplicates at the same density as described above (100 μL/well of 5 x 10^5^ cells/mL). Cells were then stimulated with 100 μL of Con A (15μg/mL), 20 μg/mL or 2 μg/mL of lysed *C*. *jejuni* (Strain A74C), or 20 μg/mL or 2 μg/mL of *Salmonella* Enteritidis OMPs. *Salmonella* Enteritidis OMPs were extracted as described previously by [38]. The 96-well plates were then incubated for 72 h, and the proliferation of MNCs was measured using MTT assay as described above.

### Statistical analysis

Student’s t-test was used to determine the effect of *Campylobacter jejuni* challenge on dependent variables. The significance level was set at (*P* < 0.05). Cage was used as an experimental unit (n = 6).

## Results

### Effect of *Campylobacter jejuni* challenge on performance parameters

There were no significant differences in FCR, BWG, or FI between the control and challenge treatments (Table 3).

**Table 3:** Effect of *Campylobacter jejuni* challenge on performance parameters.

**d14—d21**	**FCR**	**BWG (kg)**	**FI (kg)**
Control	1.064	0.444	0.542
Challenge	1.107	0.453	0.571
SEM	0.048	0.018	0.022
*P* value	0.40	0.61	0.26
**d21—d28**	**FCR**	**BWG (kg)**	**FI (kg)**
Control	1.546	0.488	0.753
Challenge	1.493	0.504	0.742
SEM	0.075	0.039	0.021
*P* value	0.51	0.70	0.61
**d28—d35**	**FCR**	**BWG (kg)**	**FI (kg)**
Control	1.601	0.475	0.759
Challenge	1.620	0.471	0.763
SEM	0.042	0.028	0.040
*P* value	0.67	0.91	0.92
**d14 –d35**	**FCR**	**BWG (kg)**	**FI (kg)**
Control	1.330	1.393	3.157
Challenge	1.327	1.422	3.207
SEM	0.014	0.053	0.077
*P* value	0.81	0.61	0.53

On d14 of age, birds were weight-matched and randomly assigned to two treatments: control and challenge. Birds were orally challenged with 0.5 mL of 2.4 x 10^8^ CFU/mL of *Campylobacter jejuni* or mock-challenged with 0.5 mL of 0.85% saline. Results were presented as mean ± SEM (n = 6).

### Effect of *Campylobacter jejuni* challenge on *Campylobacter* load in the ceca, spleen, and liver

At 7 dpi, the *C*. *jejuni* challenge treatment had a significantly higher *Campylobacter* load by 3.9, 2.5, and 0.9 log10 CFU/*g* in the ceca, spleen, and liver, respectively, when compared to the control treatment (*P* < 0.01) (Fig 1a–1c). There was a significant increase of 1.5 log10 CFU/*g* in the *Campylobacter* load in the spleen of the challenge treatment when compared to the control treatment on 14 dpi (*P* < 0.01) (Fig 1b). In general, the bacterial load in the ceca of *C*. *jejuni* challenge treatment reached around 4.9 log10 CFU/*g* on 21 dpi (Fig 1a). However, the *Campylobacter* load in the spleen and liver decreased with age in the *C*. *jejuni* challenge treatment until it reached non-detectable (ND) levels on 21 dpi (Fig 1b & 1c).

**Fig 1:** Effect of *Campylobacter jejuni* challenge on *Campylobacter* colonization kinetics in the ceca, spleen, and liver. On d14 of age, birds were weight-matched and randomly assigned to two treatments: control and challenge. Birds were orally challenged with 0.5 mL of 2.4 x 10^8^ CFU/mL of *Campylobacter jejuni* or mock-challenged with 0.5 mL of 0.85% saline. Colonization of the (a) Ceca, (b) Spleen, and (c) Liver was estimated by micro-dilutions method (CFU/g) and then log transformed to log10 CFU/g for statistical analysis. (d) *Campylobacter jejuni* in the ceca was quantified using SyBr green qPCR with primers targeting *C*. *jejuni mapA* gene. Transcript levels were reported as 40—Ct for statistical analysis. Results were expressed as mean + SEM. Non-detectable (ND). *P < 0.05; **P < 0.01 compared with control (n = 6), Student’s t-test.

### Effect of *Campylobacter jejuni* challenge on *Campylobacter jejuni mapA* gene in the ceca

At d14 (0 dpi), there were no significant differences in the *C*. *jejuni* mapA gene levels. The *mapA* gene levels were significantly higher in the *C*. *jejuni* challenge treatment on 7, 14, and 21 dpi, when compared to the control treatment (*P* < 0.05) (Fig 1d).

### Effect of *Campylobacter jejuni* challenge on serum IgY and bile IgA anti-*Campylobacter* antibodies

Day-old birds had high maternally derived IgY antibodies (OD 450 = 0.97) against *C*. *jejuni* (Fig 2a). Both treatments started with similar IgY and IgA levels at 0 dpi (Fig 2). The challenge treatment had a significant increase in IgY antibody levels on 14 and 21 dpi when compared to the control treatment (*P* < 0.05) (Fig 2a). At 7 dpi, the challenge treatment had a significant increase in specific IgA levels when compared to the control treatment (*P* < 0.01) (Fig 2b).

**Fig 2:** Effect of *Campylobacter jejuni* challenge on serum IgG and bile IgA anti-*Campylobacter* antibodies. On d14 of age, birds were weight-matched and randomly assigned to two treatments: control and challenge. Birds were orally challenged with 0.5 mL of 2.4 x 10^8^ CFU/mL of *Campylobacter jejuni* or mock-challenged with 0.5 mL of 0.85% saline. Specific (a) serum IgY and (b) bile IgA antibodies directed against *C*. *jejuni* (Strain A74C) whole cell (WC) antigens were determined by enzyme-linked immunosorbent assay (ELISA). Results were reported as mean + SEM OD 450 values. *P < 0.05; **P < 0.01 compared with control (n = 6), Student’s t-test.

### Effect of *Campylobacter jejuni* challenge on cecal tonsil CD4+ and CD8+ T lymphocytes, and CD4+:CD8+ cell ratio

At 0 dpi, the control and challenge treatments had similar percentages of CD4+ (8.23 Vs. 11.25), CD8+ T lymphocytes (2.39 Vs. 3.86), and CD4+:CD8+ cell ratio (4.45 Vs. 4.51) (Fig 3). There was a significant increase in CD4+ and CD8+ T lymphocytes in the challenge treatment on 3 dpi (*P* < 0.05) and 21 dpi (*P* < 0.01) (Fig 3a). At 14 dpi, there was a significant increase in CD8+ T lymphocytes in the challenge treatment (*P* < 0.05). There was a significant decrease in CD4+:CD8+ cell ration (1.03 Vs. 0.69) on 21 dpi (*P* < 0.05) in the challenge treatment when compared to the control treatment. A similar decrease trend in CD4+:CD8+ cell ratio (0.83 Vs 0.77) was observed in the challenge treatment on 14 dpi (*P* = 0.1) when compared to the control treatment (Fig 3b).

**Fig 3:** Effect of *Campylobacter jejuni* challenge on cecal tonsil CD4+ and CD8+ T lymphocytes, and CD4+:CD8+ cell ratio. On d14 of age, birds were weight-matched and randomly assigned to two treatments: control and challenge. Birds were orally challenged with 0.5 mL of 2.4 x 10^8^ CFU/mL of *Campylobacter jejuni* or mock-challenged with 0.5 mL of 0.85% saline. Cecal tonsils were strained to single-cell suspensions (1 × 10^6^ cells) and were incubated with PE-conjugated mouse anti-chicken CD4 and FITC-conjugated mouse anti-chicken CD8 at 1:200 dilution, and unlabeled mouse IgG at 1:500 dilution in a 96-well plate for 20 minutes. (a) CD4+ and CD8+ cells were reported as percentage of gated cells and (b) CD4+/CD8+ ratio was calculated. Results were expressed as mean + SEM. *P < 0.05; **P < 0.01 compared with control (n = 6), Student’s t-test.

### Effect of *Campylobacter jejuni* challenge on immune gene expression

At 0 and 1 dpi, both treatments had similar ceca and spleen transcript levels of the analyzed genes except for 1 dpi where there was a significant decrease in K60 mRNA levels in the spleen of the challenge treatment (Fig 4). At 3 dpi, there was a significant decrease in the mRNA levels of LITAF, K60, and CLAU-2 (*P* < 0.01) and IL-1β, iNOS, and IL-6 (*P* < 0.05) in the ceca. On the same day, a similar trend of a decrease in mRNA levels of TLR-4 (*P* = 0.06) and ZO-1 (*P* = 0.09) was observed in the ceca (Fig 5a). At 7 dpi, the ceca of the challenged birds had a significant increase in LITAF and IL-4 mRNA levels (*P* < 0.05) and a similar trend for iNOS mRNA levels (*P* = 0.07) was observed (Fig 5c). At 14 dpi, the challenged birds had a significant increase in TGF-β, IL-10, IL-1β, LITAF, TLR-4, iNOS, IL-4, and K60 mRNA levels in the spleen (*P* < 0.05) (Fig 6b). On the same day, there was a significant increase in TLR-4 mRNA levels (*P* < 0.05), and a similar increase in IL-4 mRNA levels (*P* = 0.06) in the ceca (Fig 6a). At 21 dpi, the challenged birds had a significant 2.7-fold increase in IL10 mRNA levels and a 2.4-fold increase in LITAF mRNA levels in the ceca when compared to the control treatment (*P* < 0.05) (Fig 6c).

**Fig 4:** Effect of *Campylobacter jejuni* challenge on immune gene expression in cecal tonsils at (a) 0 dpi and (c) 1 dpi, and spleen at (b) 0 dpi and (d) 1 dpi. On d14 of age, birds were weight-matched and randomly assigned to two treatments: control and challenge. Birds were orally challenged with 0.5 mL of 2.4 x 10^8^ CFU/mL of *Campylobacter jejuni* or mock-challenged with 0.5 mL of 0.85% saline. Transcript levels of genes were determined by real-time RT-qPCR. Results were expressed as the mean + SEM fold change in tissue mRNA levels in the challenge treatment as compared to the mock-challenged control treatment. *P < 0.05; **P < 0.01 compared with control (n = 6), Student’s t-test.

**Fig 5:** Effect of *Campylobacter jejuni* challenge on immune gene expression in cecal tonsils at (a) 3 dpi and (c) 7 dpi, and spleen at (b) 3 dpi and (d) 7 dpi. On d14 of age, birds were weight-matched and randomly assigned to two treatments: control and challenge. Birds were orally challenged with 0.5 mL of 2.4 x 10^8^ CFU/mL of *Campylobacter jejuni* or mock-challenged with 0.5 mL of 0.85% saline. Transcript levels of genes were determined by real-time RT-qPCR. Results are expressed as the mean + SEM fold change in tissue mRNA levels in the challenge treatment as compared to the mock-challenged control treatment. *P < 0.05; **P < 0.01 compared with control (n = 6), Student’s t-test.

**Fig 6:** Effect of *Campylobacter jejuni* challenge on immune gene expression in cecal tonsils at (a) 14 dpi and (c) 21 dpi, and spleen at (b) 14 dpi and (d) 21 dpi. On d14 of age, birds were weight-matched and randomly assigned to two treatments: control and challenge. Birds were orally challenged with 0.5 mL of 2.4 x 10^8^ CFU/mL of *Campylobacter jejuni* or mock-challenged with 0.5 mL of 0.85% saline. Transcript levels of genes were determined by real-time RT-qPCR. Results are expressed as the mean + SEM fold change in tissue mRNA levels in the challenge treatment as compared to the mock-challenged control treatment. *P < 0.05 **P < 0.01 compared with control (n = 6), Student’s t-test.

### Effect of *Campylobacter jejuni* challenge on nitric oxide production from adherent splenocyte MNCs

At 3 dpi, the challenged birds had significantly higher nitrite concentrations after LPS (54.6 Vs. 4.6 μM) and *C*. *jejuni* (72 Vs. 4 μM) *ex vivo* stimulation when compared to the control treatment (*P* < 0.05) (Fig 7). There were no significant differences in nitric oxide production levels between the control and challenge treatments at other time points (1, 7, 14, and 21 dpi) (Fig 7).

**Fig 7:** Effect of *Campylobacter jejuni* challenge on nitric oxide production from adherent splenocyte MNCs stimulated *ex vivo*. On d14 of age, birds were weight-matched and randomly assigned to two treatments: control and challenge. Birds were orally challenged with 0.5 mL of 2.4 x 10^8^ CFU/mL of *Campylobacter jejuni* or mock-challenged with 0.5 mL of 0.85% saline. Adherent splenocyte MNCs (5 x 10^4^ cells) were stimulated with 10 μg/mL of LPS or 20 μg/mL of lysed *C*. *jejuni* (CJ). After 48 h of stimulation, NO production was measuring using the Griess assay. Results were expressed as mean + SEM nitrite concentration (μM). Non-detectable (ND). *P < 0.05; **P < 0.01 compared with control (n = 6), Student’s t-test.

### Effect of *Campylobacter jejuni* on the proliferation of cecal tonsil MNCs

At 3 dpi, there was a significant suppression in T lymphocytes derived from the cecal tonsils of challenged birds when compared to the control birds after 72 h of *ex vivo* stimulation with Con A or *C*. *jejuni* (*P* < 0.05) (Fig 8a).

**Fig 8:** Effect of *Campylobacter jejuni* challenge on the proliferation of cecal tonsil *MNCs stimulated ex vivo*. On d14 of age, birds were weight-matched and randomly assigned to two treatments: control and challenge. Birds were orally challenged with 0.5 mL of 2.4 x 10^8^ CFU/mL of *Campylobacter jejuni* or mock-challenged with 0.5 mL of 0.85% saline. Cecal tonsil MNCs (5 x 10^4^ cells) were stimulated with 15 μg/mL of Con A or 20 μg/mL of lysed *C*. *jejuni* (CJ) on (a) d15 and d17 or Con A (15 μg/mL), CJ (20 μg/mL), 1:10 CJ (2 μg/mL), *Salmonella* Enteritidis (SE) OMP (20 μg/mL), or 1:10 SE OMP (2 μg/mL) at (b) 7 dpi, (c) 14 dpi, and (d) 21 dpi. The proliferation of MNCs was measured by MTT assay after 72 h of stimulation. Results were expressed as mean + SEM OD 570 values. *P < 0.05; **P < 0.01 compared with control (n = 6), Student’s t-test.

### *Ex vivo* stimulation of cecal tonsil MNCs with lysed *C*. *jejuni* (Strain A74C) or *Salmonella* Enteritidis OMPs

At 7 dpi, there was a significant suppression in the proliferation of MNCs derived from the cecal tonsils of birds in the challenge treatment when compared to the control treatment after 72 h of *ex vivo* stimulation with diluted *C*. *jejuni* (*P* < 0.05) (Fig 8b). At 14 dpi, there were no significant differences between the two treatments irrespective of the *ex vivo* stimulant (Fig 8c). At 21 dpi, there was a significant increase in the proliferation in MNCs derived from the cecal tonsils of birds in the challenge treatment when compared to the control treatment after 72 h of *ex vivo* stimulation with 1:10 diluted *C*. *jejuni* (*P* < 0.05) but not in Con A, *C*. *jejuni*, SE OMP, or diluted SE OMP stimulated MNCs (Fig 8d).

## Discussion

This study characterized the immune response of broilers to *Campylobacter jejuni* (Strain A74C). *Campylobacter jejuni* is generally considered a commensal in poultry, including broilers, and many researchers reported the bacterial isolation from a wide range of domestic poultry [10, 39]. The commensal nature of *Campylobacter* in broilers observed in our study was supported by previous studies which showed a high bacterial load in the ceca (9 log10 CFU/g), absence of pathology in *Campylobacter*-positive birds, and similar performance parameters in colonized and control birds [5, 40]. There were no significant differences in performance parameters in this study, namely FCR, BWG, and FI, between the challenge and the control treatments. Our results agree with most research studies conducted to study the effect of *Campylobacter* challenge in chickens, which showed that *Campylobacter* does not alter performance parameters and is asymptomatic in birds. However, other researchers have shown that *Campylobacter* is capable of reducing body weight and affecting performance parameters by disrupting nutrient absorption and competing for amino acids in the gut [7, 41, 42]. The different results in performance parameters seen between our study and other studies might be due to the differences in the *C*. *jejuni* isolates selected and chicken breeds used in our study, immune status, and challenge models.

In the present study, *Campylobacter jejuni* (Stain A74C) colonized the ceca of challenged birds on 7 dpi (*P* < 0.05) and persisted in the ceca until 21 dpi (d35 of age). In addition to direct plating, *Campylobacter jejuni* was quantified by qPCR targeting the *mapA* gene transcript levels. On d14 (0 dpi), there was no significant difference in *mapA* gene levels between the two treatments. However, post-challenge, *mapA* gene detection in the ceca followed the direct plating trend seen as an increase in bacterial load in challenged birds over time. *Campylobacter jejuni* was disseminated from the ceca and was detected in the spleen and liver of challenged birds with a significant *Campylobacter* load compared to the control birds (Spleen 7 dpi and 14 dpi *P* < 0.05; Liver 7 dpi *P* < 0.05). However, challenged birds cleared the *Campylobacter* load in the spleen and liver on d35 (21 dpi). Interestingly, the clearance of *Campylobacter* from the spleen and liver was accompanied by an increase in specific serum anti-*Campylobacter* IgY antibodies observed in challenged birds when compared to the control birds. Most commercial broiler flocks remain *Campylobacter*-negative until 2-wk of age. This early protection has been attributed to maternally derived antibodies [8, 43]. In our study, we observed that there were high levels of serum specific IgY maternally derived antibodies against *Campylobacter* on d0 of age confirming that early protection reported by other researchers may be due to the presence of IgY maternally derived antibodies. Bile serves a reservoir for IgA antibodies in chickens. IgA might be the most important immunoglobulin involved in mucosal immunity due to the complex it forms with the secretory component acquired from the surface of epithelial cells. This secretory component protects IgA from digestion in the gut [44]. At 7 dpi, there was a significant increase in bile specific IgA antibodies against *Campylobacter*. However, this increase in IgA levels did not affect the *Campylobacter* colonization in the ceca (4.2 log10 CFU/g). To study the effect of B cells on *Campylobacter* colonization, scientists have shown that *Campylobacter* was able to colonize the ceca of bursectomised birds concluding that humoral immunity has a limited impact on *Campylobacter* colonization in the ceca of commercial broilers [45]. Researchers have demonstrated that *Campylobacter* is able to disseminate to internal organs, including the spleen, liver/gallbladder, thymus, and bursa of Fabricius, after challenge via the oral route [9]. Interestingly, prior to bacterial dissemination to internal organs observed at 7 dpi, *Campylobacter*-challenged birds where immunosuppressed at 3 dpi. This immunosuppression was seen as a suppression in cecal tonsil MNCs stimulated with either Con A (indicating that it is a T cell suppression (3 dpi)), lysed *C*. *jejuni* (3 dpi), or lysed and diluted *C*. *jejuni* (7 dpi). In addition to the suppression in cecal tonsil MNCs’ proliferation, a significant decrease in gene expression at 3 dpi was observed for both immune genes (LITAF, K60, IL-1β, iNOS, IL-6, and TLR-4) and tight junction proteins (CLAU-2 and ZO-1). Other researchers have compared the immune response of broilers to *Campylobacter* versus *Salmonella* challenge and have shown that unlike *Salmonella*, *C*. *jejuni* challenge significantly downregulated the antimicrobial peptide gene expression 6 h post infection [46]. The immune suppression of MNCs, cytokines, and tight junction proteins seen in our study might explain the high bacterial colonization in the ceca and the bacterial dissemination from the gut to internal organs in broilers. At 14 dpi, there was a significant upregulation in both pro- and anti-inflammatory cytokines in the spleen. This upregulation in both pro- and anti-inflammatory cytokines suggests that a balanced Th1 and Th2 immune response might explain the absence of pathology in *Campylobacter*-challenged birds.

Nitric oxide production is critical for vasodilation, neurotransmission, and host pro-inflammatory immune response against pathogens and tumors. Nitric oxide production is mediated by Nitric Oxide Synthase (NOS). In chickens, nitric oxide is mainly secreted by macrophages and monocytes and is induced by intracellular pathogens, some tumors, LPS, and IFN-γ [47]. In the present study, mononuclear cells derived from the spleen of *Campylobacter jejuni*-challenged birds 3 dpi had a significant increase in nitrite concentrations, when compared to MNCs from the control birds, after 48 h of *ex vivo* stimulation with *Salmonella enteritidis* LPS or the homologous lysed *C*. *jejuni*. In addition, an upregulation in pro-inflammatory genes such as LITAF, IL-1β, and iNOS in either the spleen, ceca, or both was observed in the *C*. *jejuni* challenged birds. These data present further evidence of bacterial dissemination to internal organs, seen in our study and other studies, and is in agreement with other studies that have shown that *Campylobacter* is not purely a commensal but that chickens mount a pro-inflammatory immune response post-infection [6, 11, 46]. *In vitro* and *in vivo* experiments showed that *Campylobacter* is usually recognized by TLR4 and TLR21 [48, 49]. In our study, we looked at TLR-4 and observed that *C*. *jejuni* challenge decreased the mRNA levels of TLR-4 in the ceca 3 dpi, and upregulated TLR-4 in both the ceca and spleen 14 dpi.

In many species, including chickens, mice, and humans, CD4+:CD8+ cell ratio is an indicator of immune competence [47, 50, 51]. In general, a CD4+:CD8+ cell ration that is higher than 1, reflecting a higher percentage of CD4+ cells relative to CD8+ cells, is observed in healthy individuals. Age, dietary treatment, breed, and disease status, are factors reported to change the CD4+:CD8+ cell ratio in chickens [52–55]. In our study, we observed that *C*. *jejuni* challenge increased significantly CD4+ and CD8+ T lymphocytes 3 and 21 dpi and CD8+ cells on 14 dpi. The CD4+:CD8+ cell ratio was decreased numerically (0.83 Vs. 0.77) at 14 dpi (*P* = 0.1) and significantly (1.03 Vs. 0.69) at 21 dpi (*P* < 0.05) when comparing *C*. *jejuni*-challenged birds to the control. This indicates that the increase in CD8+ cells was of greater magnitude when compared to the increase in CD4+ cells. At 21 dpi, cecal tonsil MNCs derived from the challenged treatment had a significantly higher antigen-specific proliferation when compared to MNCs from the control treatment after *ex vivo* stimulation with the diluted lysed *C*. *jejuni*. These data support our flow cytometry data which showed a significant increase in both CD4+ and CD8+ T-lymphocytes 21 dpi in *C*. *jejuni*-challenged birds. In addition, 21 dpi, a significant upregulation in LITAF and IL-10 was observed. Our observation of IL-10 upregulation in *C jejuni* challenged birds agrees with other researchers who showed that *Campylobacter* persistence and the absence of pathology in challenged birds was associated with an upregulation in IL-10 in challenged birds [6]. Many researchers speculate that regulatory T cells play a major role in orchestrating the commensal nature of *Campylobacter* in chickens [6, 56]. Avian regulatory cells suppress other immune cells through both a contact-dependent mechanism and a contact-independent mechanism (mediated by the production of IL-10 and TGF-β) [57]. Other researchers attributed the commensal nature of *Campylobacter* to its ability to induce a Th17 response that restricts the bacterial colonization to the intestine [58]. Other studies focused on understanding the colonization factors of *C*. *jejuni* strains and concluded that these factors could be responsible for the commensal nature of *Campylobacter* in chickens and its infectious nature in humans [59, 60]. In this study we show proinflammatory, anti-inflammatory, and regulatory cytokines were expressed after *Campylobacter jejuni* challenge and agrees with findings by other researchers [58].

In conclusion, our study shows that *Campylobacter jejuni* (Strain A74C) colonized the ceca of broilers at a high level and disseminated to the spleen and liver. Over time, *Campylobacter jejuni* persisted in the ceca, but was cleared from the spleen and liver accompanied by a significant increase in specific serum IgY antibodies. Our study demonstrated that *Campylobacter jejuni* can induce an inflammatory response in chickens. The Th1 immune response was evident in the production of NO from the adherent splenocytes, the upregulation of different pro-inflammatory cytokines at different timepoints in the spleen and cecal tonsils, and the increase in CD8+ cells. However, the upregulation in anti-inflammatory and regulatory cytokines, T lymphocyte proliferation suppression 3 dpi, the increase in CD4+ cells, and the increase in specific serum IgY levels suggest that *C*. *jejuni* also induced a Th2 immune response. Therefore, the balance between the Th1 and Th2 immune responses against *C*. *jejuni* might explain the bacterial persistence in the ceca and the absence of pathology in *Campylobacter*-challenged birds. Future studies directed at studying the T lymphocyte subpopulations are needed to elucidate the pivotal role that T lymphocytes play in the persistence of *Campylobacter* in the ceca and will be valuable for developing successful interventions.
